The article "Study on the Correlation Factors of Tumour Prognosis after Intravascular Interventional Therapy" was retracted in 2023. Reasons: suspected computer-generated content; unreliable results or conclusions; lack of ethics approval or compliance; missing or withdrawn patient consent.

# Study on the Correlation Factors of Tumour Prognosis after Intravascular Interventional Therapy

**DOI:** 10.1155/2021/6940056

**Published:** 2021-10-27

**Authors:** Lei Zheng, Hua Feng, Limin Yin, Jun Wang, Wei Zhou, Sunin Tang, Mingming Li

**Affiliations:** ^1^Taizhou Hospital of Traditional Chinese Medicine, Taizhou Jiangsu 225300, China; ^2^Taixing People's Hospital, Taizhou, Jiangsu 225400, China; ^3^First Affiliated Hospital of Soochow University, Suzhou Jiangsu 215000, China

## Abstract

Noninvasive or minimally invasive interventional surgery was selected, and the complications were less and had no significant impact on the quality of life of patients. Tumour patients are often accompanied by cerebrovascular diseases, metabolic diseases, and other basic diseases, which more or less adversely affect the surgical efficacy of tumour. In this paper, endovascular remobilization was used to treat tumour; the basic condition of patients before operation and the interventional operation plan were introduced. Through the analysis of clinical data and prognosis evaluation results of tumour patients receiving intravascular interventional therapy, the patients were divided into good prognosis group and poor prognosis group according to the modified Rankin scale score at discharge. The relationship between gender, age, history of hypertension, tumour width, tumour size, preoperative Hunt-Hess grade, interventional surgery method, and prognosis related to intravascular interventional therapy was explored. The results showed that intravascular interventional therapy for tumour patients can obtain a good prognosis, which provides a reference for the future preoperative assessment of treatment risk and possible prognosis and provides a theoretical basis for the formulation of treatment plan to improve prognosis.

## 1. Introduction

Combined tumour therapy includes surgery, radiotherapy, and chemotherapy. With the development of advanced technologies such as imaging, microcatheters, and stents, interventional therapy is providing new treatments for diseases that were previously untreatable or ineffective. Tumour therapy has entered the noninvasive or minimally invasive era. The purpose of digital subtraction angiography intravascular interventional therapy of tumour is to improve the therapeutic effect of local tumour and overcome the disadvantages of traditional treatment such as intravenous systemic chemotherapy, such as adverse reactions, radiation damage, and severe injury. Preoperative tumour interventional therapy can reduce tumour staging, improve surgical resection rate and survival rate, and reduce postoperative recurrence and metastasis. Interventional therapy for patients with advanced cancer can improve the quality of life and prolong the overall survival time of patients with cancer [1–3]. Therefore, interventional therapy has become one of the important means of comprehensive tumour therapy. However, there are still many weak links in the relevant basic and clinical research, especially the study of pharmacokinetics.

The article "Study on the Correlation Factors of Tumour Prognosis after Intravascular Interventional Therapy" was retracted in 2023. Reasons: suspected computer-generated content; unreliable results or conclusions; lack of ethics approval or compliance; missing or withdrawn patient consent.

With the development of medicine, interventional surgery has been applied more and more widely, not only in medical treatment, but also in surgery. Interventional therapy is appropriate for patients with severe bleeding due to trauma or whose tumours are unsuitable for major surgery. The intervention not only has less trauma and bleeding, but also recovers quickly. As long as there is a risk of surgery, interventional surgery is the same; different primary disease interventional complications are also different. The operation of interventional surgery has been greatly developed, so it has become a major minimally invasive surgical therapy not only applied to the back circulation but also widely applied to tumours. It has been recognized and accepted by the majority of patients for its accurate surgical efficacy, high success rate, and good prognosis. By adopting elastic yellow ring or stent-assisted embolization experience and clinical data, interventional embolization is safe and has a good curative effect of new treatments [4, 5], especially for some tumours that be treated with open surgical operation or difficult high risk patients, intravascular interventional embolization has become a preferred therapy. Interventional surgery is a modern, high-tech, and minimally invasive treatment method, which is introduced into the body by using professional catheter or guide wire and other instruments, combined with medical imaging equipment, to judge and treat diseases. Interventional therapy is an advanced science and technology developed in recent years. It has the advantages of small trauma and effective and rapid recovery by interventional therapy on the premise of no operation. Interventional therapy is now widely used. In the past, many operations that cannot be done clinically or are very difficult can be operated simply and effectively through interventional surgery. Now, it is mostly used for tumours, cardiovascular and cerebrovascular diseases, nervous system, gynaecological problems, all kinds of bleeding, stones, and so on. Especially in liver cancer and liver haemangioma effect is very significant; in addition to myocardial infarction this effect is very significant.

As a relatively new treatment method, the prognosis of intravascular interventional therapy for IA has attracted much attention. Under the guidance of imaging equipment, doctors send a special catheter to the tumour's supplying artery and then inject embolization material through the catheter to completely embolize the tumour's supplying artery. B. Taslakian et al. studied the related factors that may affect the prognosis of invasive surgery, including the basic information of patients, such as gender, age, etc., which are thought to be associated with tumour incidence that is closely related to the basic diseases such as hypertension, tumour size, tumour related specific morphological features, such as neck width, and different ways of interventional surgery, the patient's clinical status classification, etc. [5]. At present, prognostic factors have not been clearly defined. O. Sutte et al. listed simple coil embolization, preoperative Hunt-Hess grade III-IV, and tumour diameter >10 mm as independent risk factors affecting the prognosis of tumour patients after endovascular intervention, while age, sex, underlying diseases, tumour neck width, and other indicators had no significant correlation with prognosis [6]. Lee et al. believe that Hunt-Hess grade of patients, tumour location and size, and other factors are independent risk factors affecting interventional efficacy and postoperative tumour rupture [7]. L. Wang et al. believe that most patients are complicated with atherosclerosis, arteriosclerosis, and other vascular diseases and are more prone to mini-ischemia [8]. Chang study showed that aneurysm diameter ≥7 mm and tumour neck size ≥4 mm were significantly correlated with symptomatic cerebral microischemia and DWI (+). The size and shape of aneurysms are also associated with increased thromboembolic events detected by Diffusion Weighted Imaging (DWI) [9]. Larger or wide-necked aneurysms usually require more coils or the use of double catheters, balloon reconstruction, or stent-assisted techniques, theoretically increasing the risk of thromboembolic complications. However, different research data support that the ratio of tumour length to tumour neck width (AR) and hypertension are included as prognostic factors. L. Tselikas pointed out that, due to different locations, the prognosis of anterior and posterior circulation tumours is significantly different after interventional therapy [10]. However, most previous studies related to prognostic factors involve multisite tumours and lack pertinence to the location of tumours.

The article "Study on the Correlation Factors of Tumour Prognosis after Intravascular Interventional Therapy" was retracted in 2023. Reasons: suspected computer-generated content; unreliable results or conclusions; lack of ethics approval or compliance; missing or withdrawn patient consent.

## 2. Data and Methods

### 2.1. Preoperative Data

In this study, clinical data of tumour patients undergoing intravascular intervention therapy in a hospital were selected, including age, smoking history, hypertension history, diabetes history, hyperlipidemia, aneurysm location and size, whether it was a wide-necked aneurysm, stent use, platelet suppression 1 day before surgery, and operation duration. All patients were diagnosed with intracranial aneurysm by CT angiography (CTA) and digital subtraction angiography (DSA). Magnetic Resonance Imaging (MRI) of the head was completed 3 days after surgery. All signed informed consent forms: patients with systemic infectious diseases, severe organ dysfunction, and other surgical contraindications; dissecting aneurysm, pseudoaneurysm and intracranial multiple aneurysm; pregnancy with intracranial aneurysm; intracranial and extracranial artery stenosis; intraoperative acute thrombosis and intraoperative aneurysm rupture. After admission, the patient was closely monitored in the neurological care unit, with absolute bed rest, appropriate sedation, and analgesia treatment, and stool was kept unapparent. Blood pressure was regulated to keep systolic pressure within 160 mmHg, while ensuring that the mean arterial pressure is higher than 90 mmHg. According to the patient's condition, drugs to relieve cerebral vasospasm, dehydration to reduce cranial pressure, lumbar puncture cerebrospinal fluid replacement, lateral ventricle drainage, and other treatments were used, and further interventional therapy was performed after preoperative examination was completed and the condition was stabilized [11]. The preoperative procedure is shown in Figure 1.

### 2.2. Interventional Therapy

Simple core embolization, double microcatheter remobilization, or stent-assisted core-remobilization was selected according to the patient's condition, the situation of pulsar tumour, and the patient's willingness. During the operation, the patient was placed in the supine position. After tracheal intubation and general anaesthesia, the puncture site with the most obvious pulse 1.5 cm below the right inguinal ligament was selected as the puncture site. After routine skin disinfection for three times, sterile towel was covered. After percutaneous femoral artery puncture and catheter sheath placement, the catheter was guided from the femoral artery all the way up to the internal carotid artery. Microguide wires and microcatheters were used in the operation, and the appropriate working angle was selected in combination with the 3D reconstruction image during the operation. Remobilization with simple coil is to send a microcatheter to the tumour cavity under the guidance of a microguide wire and to deliver a certain number of microcoils through the microcatheter to fill according to the tumour size and shape nad width of the tumour neck and the parent artery.

For relatively broad neck tumours or broad neck tumours with difficult stent placement, double microcatheter technology was adopted. Under the operation of two microcatheters, spring coils were, respectively, transported into the tumour cavity, and remobilization effect was achieved by winding the spring coils together into a basket. Stent-assisted coiling remobilization (SAC) is to perform coiling remobilization in the tumour cavity on the basis of placing stents in the tumour neck with absolute or relatively wide neck by microcatheter, so as to close the tumour neck and avoid coiling displacement [12]. The therapeutic objective and ideal state of all treatment methods are that there is no development in the tumour and there is spring coil tamping in the neck of the tumour immediately after treatment.

The article "Study on the Correlation Factors of Tumour Prognosis after Intravascular Interventional Therapy" was retracted in 2023. Reasons: suspected computer-generated content; unreliable results or conclusions; lack of ethics approval or compliance; missing or withdrawn patient consent.

During the operation, the patient's whole body heparin was maintained, and high pressure heparin saline was administered to continuously flush the lumen to avoid thrombosis in the lumen guided by the catheter. It was expected that patients using stents would be given clopidogrel tablets 75 mg/d and enteric-coated aspirin tablets 100 mg/d 3 days before surgery. In case of emergency, preoperative disposable clopidogrel tablets 300 mg and enteric-coated aspirin tablets 300 mg were used.

The above operations are performed by skilled people. 24 hours after the operation, strict ECG monitoring, and give anticerebral vasospasm, anti-inflammatory, fluid replacement, expansion, dehydration, and other treatments. After 3 days of subcutaneous injection of low molecular weight heparin sodium, patients were treated with oral clopidogrel 75 mg/d and enteric-coated aspirin 100 mg/d for 6 months and then maintained with enteric-coated aspirin 100 mg/d or clopidogrel 75 mg/d.

All interventional procedures were performed by the same neurosurgeon via femoral artery approach under general anaesthesia. A complete set of thromboelastography (AA% and ADP%) was completed for all patients 1 day before surgery. Both patients received dual antiplatelet therapy (aspirin 300 mg and clopidogrel 300 mg) 2 hours before surgery. After successful general anaesthesia, heparinization was performed on the whole body, the dosage was 1 mg/Kg, and the dosage was reduced to 50% of the previous dosage 1 hour later until the reduction was maintained at 10 mg/hour. Procaine and heparin were given at the end of the operation if only coiling embolization of the tumour was performed. If stent-assisted embolization of the tumour is used intraoperatively, no heparin is obtained. After the operation, the coagulation image was examined immediately. If the coagulation result reached the indication of blood transfusion, plasma was given to improve the coagulation function. If stent-assisted embolization of tumour is used, subcutaneous anticoagulant injection of low molecular weight heparin should be used according to the preoperative inhibition of TEG platelet [13]. If aspirin and/or clopidogrel resistance, low liver 4000IU Q12 h is given. If both aspirin and clopidogrel were sensitive, the liver was lower than 2000IU q12 h. After 3 days, it was changed to double therapy. If no stents were used, hypohepatic and double-antitumor therapy was not used after surgery. The procedure of interventional surgery is shown in Figure 2.

The article "Study on the Correlation Factors of Tumour Prognosis after Intravascular Interventional Therapy" was retracted in 2023. Reasons: suspected computer-generated content; unreliable results or conclusions; lack of ethics approval or compliance; missing or withdrawn patient consent.

### 2.3. Prognostic Data Collection

In this study, the relevant data of the included patients during outpatient, inpatient, or telephone follow-up 6 months to 1 year after surgery were collected, and the prognosis of the patients was evaluated according to the scores of the modified Rankin scale, as shown in Table 1. Disability and death mentioned in the criteria are related to responsible tumours, excluding heart disease, cirrhosis, and other factors. The patients were grouped according to the mRS score, with 0–2 points included in the good prognosis group and 3–6 points included in the poor prognosis group [14, 15].

### 2.4. Statistical Method

SPSS21 statistical software was used for statistical analysis. The data of normal distribution were represented by mean ± standard deviation, and the data of nonnormal distribution was represented by median ± quartile interval. The counting data are expressed by frequency and percentage. University analysis was performed on indicators that may affect prognosis, including gender, age, history of hypertension, tumour neck width, tumour diameter size, preoperative Hunt-Hess grade, and interventional surgery. The continuous variables were converted into classified variables, and Pearson chi-square test (sample size *n* ≥ 40 and theoretical frequency *T* ≥ 5) or corrected chi-square test (*n* ≥ 40, 1≤*T* ≤ 5) or Fisher exact probability method (*n* < 40 or *T* < 1) was used. *P* < 0.05 was considered statistically significant. The factors with statistical significance in univariate analysis were further analyzed by multivariate analysis: logistic regression analysis; *P* < 0.05 was considered statistically significant [16, 17].

## 3. Result

### 3.1. Basic Information of the Patient

A total of 63 patients, including 23 males and 40 females, were enrolled in the Body Mass Index (BMI) study. The investigation and analysis of patients took into account the factors of previous pathological history, hypertension, smoking history, and diabetes. Thirty-one patients had a history of hypertension, 22 had a history of diabetes, and 21 had a history of smoking. The highest age was 62 years, the lowest age was 20 years, and the average age was 57.3 ± 10.3 years. BMI ranged from 36.3 to 16.7, with a mean value of 24.0 ± 3.3. The statistical results are shown in Figure 3.

The article "Study on the Correlation Factors of Tumour Prognosis after Intravascular Interventional Therapy" was retracted in 2023. Reasons: suspected computer-generated content; unreliable results or conclusions; lack of ethics approval or compliance; missing or withdrawn patient consent.

Sixty-three patients had a total of 68 tumours, of which 60 were treated with interventional therapy and 8 were untreated. Among them, there were 66 responsible tumours (as shown in Table 2): 23 anterior traffic tumours, 5 anterior brain tumours, 16 brain tumours, 18 intracranial tumours of internal carotid artery, and 14 posterior traffic tumours.

### 3.2. Interventional Therapy

Among the 63 cases of anterior circulation responsible tumours receiving intravascular interventional therapy, 43 cases received simple coiling embolization therapy, 1 case received double microcatheter embolization therapy, and 19 cases received stent-assisted coiling embolization therapy. The distribution of interventional therapy methods is shown in Figure 4.

### 3.3. Postoperative Angiography and Clinical Results

The total immediate dense embolization rate was 80.2%, and the rate of subcomplete and incomplete embolization was 17.6%. Because the follow-up time of each patient is not consistent, the follow-up embolization degree has no statistical value and was not analyzed. In terms of clinical results, one patient with superior cerebella artery tumour frequently vomited after stent-assisted embolization, and the second angiography showed that the parent artery was preserved without thrombosis. Another patient with superior cerebella artery tumour had blurred vision due to parent artery occlusion. 1 case of posterior inferior cerebella artery dissection tumour underwent stent-assisted coiling embolization with reduced muscle strength in the left limb. A patient with a large middle cerebral artery tumour undergoing parent artery occlusion showed reduced muscle strength in the left limb after surgery. Postoperative rebreeding occurred in 2 cases, including 1 in inferior posterior cerebella artery and 1 in middle cerebral artery, and parent artery occlusion was performed in both cases. Microischaemic lesions occurred in 34 of the 63 patients. The statistical results are shown in Figure 5.

### 3.4. Prognostic Factor Analysis

#### 3.4.1. Relationship between Age, Sex, Hypertension, and Prognosis

The age of patients was divided into three segments by 40 and 60. In the intravascular intervention group, the poor prognosis rate of patients <40 years old was 6.00%, that of patients 40–59 years old was 7.89%, and that of patients ≥60 years old was 30.00%. There was no statistical significance between the poor prognosis rates. In the vascular intervention group, the poor prognosis rate of male patients was 13.16%, and the poor prognosis rate of female patients was 6.67%. There was no statistical significance between the poor prognosis rates. In the vascular intervention group, the poor prognosis rate of patients with hypertension history was 19.36%, and that of patients without hypertension history was 4.48%, and the difference between the poor prognosis rates was statistically significant. The relationship between age at onset, sex, hypertension, and prognosis is shown in Figure 6.

The article "Study on the Correlation Factors of Tumour Prognosis after Intravascular Interventional Therapy" was retracted in 2023. Reasons: suspected computer-generated content; unreliable results or conclusions; lack of ethics approval or compliance; missing or withdrawn patient consent.

Statistical analysis showed that there was no statistically significant difference in prognosis between male and female patients, so gender difference was not an independent risk factor affecting the prognosis of tumour interventional therapy. Endovascular interventional therapy is a minimally invasive surgery, which has less tissue trauma and surgical impact on patients than craniotomy and clipping surgery, and the endurance of the elderly is relatively improved. Elderly patients can give priority to endovascular interventional therapy, and old age is not an absolute contraindication for interventional surgery.

Hypertension is regarded as a common risk factor by most scholars. Long-term hypertension can lead to damage of vascular endothelial cells, apoptosis of vascular smooth muscle cells in the media, rupture and disappearance of elastic fibbers, and gradual thinning of vascular walls. On this basis, changes in hemodynamics promote the formation of lesions. High vascular wall shear stress and high blood flow velocity have a strong blocking effect on local tumour thrombosis. Meanwhile, hypertension can also affect the hemodynamic parameters and increase the shear force of the vascular wall at the intracranial artery bifurcation, causing damage to the vascular wall and aggravating the condition of intracranial aneurysm. In the process of intravascular interventional therapy, the lesion site cannot be thromboses and the healing of the tumour is hindered. In addition, the high speed blood flow can also lead to microspring compression and increase the risk of recurrence, which is unfavourable before and after tumour [18, 19]. Avoiding large fluctuations in blood pressure can prevent exacerbation and progression of the disease, and even patients with hypertension can obtain a good prognosis.

#### 3.4.2. Relationship between Preoperative Hunt-Hess Grade, CT-Fisher Grade, and Prognosis

In the endovascular intervention group, the prognostic rates of grade I, II, III, and IV patients were 0%, 9.09%, 8.33%, and 80.00%, respectively, with statistically significant differences. In the vascular intervention group, the preoperative CT-Fisher grade poor prognosis rate of grade I was 0.00%, grade II was 1.69%, grade III was 8.33%, and grade IV was 13.64%, with statistically significant differences in the poor prognosis rate. The relationship between preoperative Hunt-Hess grade, CT-Fisher grade, and prognosis was shown in Figure 7.

The article "Study on the Correlation Factors of Tumour Prognosis after Intravascular Interventional Therapy" was retracted in 2023. Reasons: suspected computer-generated content; unreliable results or conclusions; lack of ethics approval or compliance; missing or withdrawn patient consent.

Hunt-hess grade is an objective index reflecting the clinical status of patients, which evaluates patients according to headache degree, meanings irritation, consciousness state, nervous system function state, etc. [18]. There was no statistically significant difference in prognosis among patients with different Hunt-Hess grades. It was considered that some patients with high Hunt-Hess grade were not included in this study because of their serious condition and high risk of intervention therapy, and they died before receiving treatment or finally decided to receive conservative treatment, give up treatment or surgical clamping treatment, or transferred to hospitals according to the wishes of their families. Therefore, in this study, the number of cases with lower Hunt-Hess grade was significantly more than those with higher Hunt-Hess grade, and there was a certain selection bias. Although Hunt-Hess grade IV and V cases were combined into one group for statistical analysis, the results still showed no statistically significant difference in prognosis. In addition, the intervention before the operation, to stabilize their condition, provides the operation conditions on the Hunt-Hess rank higher in patients with lumbar puncture cerebrospinal fluid replacement, lateral ventricle drainage, and other treatments; the treatment operation to some extent reduced the degree of hydrocephalus, relieved the intracranial pressure, and dredged the cerebrospinal fluid pathway, a positive influence on the prognosis of patients. Therefore, in this study, the rate of poor prognosis did not increase with the increase of Hunt-Hess grade, and no positive results were obtained by statistical analysis.

#### 3.4.3. Relationship between Tumour Size, Tumour Width, and Prognosis

Figure 8 shows the relationship between tumour size, tumour width, and prognostics in enrolled patients. According to the results of Fisher's exact probability test, it was believed that the difference of prognosis among different tumour sizes and widths was statistically significant.

Tumour size is considered to be an independent risk factor for postoperative ischemic events. Thrombosis is more likely to occur in large aneurysms, making it difficult for the spring coil to fill the area occupied by the thrombus, and the residual cavity will be exposed and enlarged after thrombus dissolution, leading to aneurysm recurrence. In addition, oversized aneurysms may also have the problem of space occupying. Even if the space occupying effect caused by blood pulsation is relatively reduced after complete embolization, the aneurysm volume does not change significantly after embolization, and the space occupying effect of the tumour itself is not relieved, which can still cause clinical symptoms. The tumour diameter <7 mm was more prone to intraoperative rupture during endovascular therapy. Tumours larger than 7 mm had a higher incidence of thromboembolic events, but tumour size had no significant effect on intraoperative rupture. Statistical analysis showed that there was a statistically significant difference in prognosis between tumour size <7 mm and tumour size >7 mm, and tumour size >7 mm was a risk factor for poor prognosis.

The article "Study on the Correlation Factors of Tumour Prognosis after Intravascular Interventional Therapy" was retracted in 2023. Reasons: suspected computer-generated content; unreliable results or conclusions; lack of ethics approval or compliance; missing or withdrawn patient consent.

Tumour neck width and tumour body neck ratio (AR) are important indexes to reflect the geometric characteristics of tumour. The tumour neck size has a controlling effect on the eddy current velocity in the tumour cavity. Wide-neck tumours usually have larger blood flow and complex stress gradient, which affects the filling effect of spring coil [19]. Therefore, the treatment of wide-neck tumours is relatively difficult. Related studies have found that broad neck tumours show a lower complete occlusion rate in both immediate postoperative angiography and follow-up angiography [20], and broad neck tumours have a higher decimalization rate than narrow neck tumours. With the progress of embolization technology and materials, the problems such as the insertion of tamped spring coil into the parent artery through a wide neck can be solved, and even wide-necked aneurysms can obtain a relatively ideal effect [21].

Tumour diameter, tumour neck width, and multiple tumours are risk factors for recurrence of intracranial aneurysms treated by intravascular intervention. The tumours with larger diameter were more irregular, and the tamping degree of the tumour neck with larger width was lower, so recurrence was easy to occur. In addition, thrombus is more common in tumour lumen in patients with large tumour diameter, and it is difficult to completely occupy part of the space of thrombus in the process of embolization of microspring coil. With the absorption of thrombus in tumour lumen, it is easy to cause the expansion of residual lumen and relapse. Patients with multiple tumours have more tumours, more complex disease, and more difficult intravascular interventional therapy, so the prognosis is poor and the risk of recurrence is greater.

### 3.5. Single-Factor Analysis

Univariate analysis showed that patients with a history of hypertension, large tumour diameter, clopidogrel resistance, and stent-assisted embolization had a higher incidence of postoperative microischemia. Age, smoking history, diabetes history, hyperlipidemia, aspirin resistance, tumour neck size, tumour location, and surgical duration were not statistically different between the two groups. The Chi-square test and Fisher's exact probability method were used in the univariate analysis, as shown in Table 3. Aneurysm size, aneurysm morphology, aneurysm neck morphology, aneurysm treatment, aneurysm embolization degree, follow-up time, and other factors are related to aneurysm recurrence. *P* < 0.05 was considered as statistically significant.

The article "Study on the Correlation Factors of Tumour Prognosis after Intravascular Interventional Therapy" was retracted in 2023. Reasons: suspected computer-generated content; unreliable results or conclusions; lack of ethics approval or compliance; missing or withdrawn patient consent.

### 3.6. Multiple-Factor Analysis

Multivariate binary logistic regression analysis was conducted for the above two statistically significant indicators, as shown in Figure 9. The results showed that tumour size and interventional surgery method were the influencing factors for the prognosis of tumour interventional therapy. Tumour size > 7 mm and stent-assisted embolization are independent risk factors for the prognosis of patients with anterior circulation rupture. The risk of poor prognosis in patients receiving stent-assisted embolization was 4.172 times that of patients receiving non-stent-assisted embolization. The risk of poor prognosis in patients with <7 mm tumour was 0.035 times that in patients with >7 mm tumour, respectively.

The essence of the tumour lies in the local lesion of the arterial wall of the parent artery. Both stent-assisted embolization and non-stent-assisted embolization are mainly for the filling of the tumour cavity, while the treatment of the parent artery is neglected. The application of stents can effectively increase the density of tumour embolization and reconstruct the parent artery wall to surround the tumour neck. Stents improve hemodynamics and thus promote endometrial hyperplasia to cover the neck of the tumour. Multivariate logistic regression analysis showed that stent-assisted embolization had a 4.172-fold higher risk of poor outcome than non-stent-assisted embolization. In the process of stent-assisted embolization, the control and operation of stents are complicated. Once there is poor stent adherence and resistance to antiplatelet aggregation drugs, it is easy to induce platelet aggregation, promote stent thrombosis, and increase the incidence of cerebral infarction. On the one hand, choosing the stent with appropriate radial force and avoiding stimulating endothelial proliferation can reduce the chance of stinting stenosis. On the other hand, preoperative and postoperative ant platelet therapy should not be ignored. Therefore, in clinical work, the sensitivity of patients to ant platelet drugs should be well grasped, and individualized ant platelet therapy should be achieved, so as to maximize the advantages of stent-supported therapy.

The article "Study on the Correlation Factors of Tumour Prognosis after Intravascular Interventional Therapy" was retracted in 2023. Reasons: suspected computer-generated content; unreliable results or conclusions; lack of ethics approval or compliance; missing or withdrawn patient consent.

## 4. Conclusion

Endovascular interventional therapy is a minimally invasive surgery, which has less tissue trauma and surgical impact than craniotomy clipping surgery. In this paper, endovascular embolization was used to treat tumour; the basic condition of patients before operation and the interventional operation plan were introduced. Through the analysis of clinical data and prognosis evaluation results of tumour patients receiving intravascular interventional therapy, the patients were divided into good prognosis group and poor prognosis group according to the modified Rankin scale score at discharge. The relationship between gender, age, history of hypertension, tumour width, tumour size, preoperative Hunt-Hess grade, interventional surgery method, and prognosis related to intravascular interventional therapy was explored. Conclusion: tumours >7 mm are a risk factor for poor prognosis. Age, sex, history of hypertension, tumour neck width, and preoperative Hunt-Hess grade were not independent risk factors affecting the prognosis of interventional therapy for tumours with anterior circulation rupture. The prognosis of tumour after intravascular intervention was related to the age, Hunt-Hess grade, and hypertension. The recurrence of the disease is related to the patient's age, Hunt-Hess grade, diabetes, hypertension, tumour diameter, tumour neck width, surgical methods, and embolization. Clinical attention should be paid to the influence of these factors, and corresponding measures should be taken to reduce the recurrence rate and improve the prognosis. Further studies are needed to determine whether preoperative control of blood pressure levels will reduce the incidence of microthromboembolic complications.

## Figures and Tables

**Figure 1:** Preoperative flowchart.

**Figure 2:** Flowchart of interventional surgery.

**Figure 3:** The basic situation of the patient statistical graph. Basic information of tumour.

**Figure 4:** Distribution of interventional therapy.

**Figure 5:** Single-factor analysis diagram.

**Figure 6:** Patient age, sex, and prognosis diagram analysis.

**Figure 7:** Diagram of relationship between preoperative Hunt-Hess grade, CT-Fisher grade, and prognosis.

**Figure 8:** The relationship between tumour size, tumour width, and prognosis in patients.

**Figure 9:** Multivariate binary logistic regression analysis.

**Table 1:** mRS scoring criteria.

Scale of marks		
Project	Scope	Score
Age	≤40	0
	41–50	1
	51–69	2
	≥70	3

NIHSS scores	0–4	0
	5–9	1
	10–15	2
	>15	3

Defect of field vision	—	2
Decreased level of consciousness	—	3
The onset lasts more than 3 hours	—	2

The article "Study on the Correlation Factors of Tumour Prognosis after Intravascular Interventional Therapy" was retracted in 2023. Reasons: suspected computer-generated content; unreliable results or conclusions; lack of ethics approval or compliance; missing or withdrawn patient consent.

**Table 2:** Responsible for the location of the tumour distribution.

Position	Number of cases	Percentage rate (%)
Anterior communicating artery	23	34.85
Anterior cerebral artery	5	7.58
Middle cerebral artery	16	24.24
ICA	8	12.12
Posterior communicating artery	14	21.21

**Table 3:** Univariate analysis of relationship statistics.

Element	*X* ^2^	*P*
Age	1.303	0.075
Gender	0.526	0.468
Hypertension	3.982	0.056
Hunt-Hess	0	0.001
CT-Fisher	0	0.001
Tumours in diameter	0	0.002
Tumour neck width	0.987	0.388

## Data Availability

The data used to support the findings of this study are available from the corresponding author upon request.
